# An Unusual Variational Anatomy of the Medial Circumflex Femoral Artery: A Case Report of a Post-catheterization Femoral Arteriovenous Fistula

**DOI:** 10.7759/cureus.6734

**Published:** 2020-01-22

**Authors:** Yohei Yamamoto, Hidetoshi Uchiyama, Masahiro Onuki

**Affiliations:** 1 Department of Vascular Surgery, Tsuchiura Kyodo General Hospital, Tsuchiura, JPN

**Keywords:** medial circumflex femoral artery, variation, arteriovenous fistula, cardiac catheterization, femoral access

## Abstract

The medial circumflex femoral artery (MCFA) typically presents as a major branch of the profunda femoris artery or it can also directly originate from the common femoral artery. Many anatomical variations of the MCFA have been described due to their clinical significance. We herein report a case of an unusual anatomical variation of the MCFA crossing anterior to the femoral vein that led to iatrogenic arteriovenous fistula formation after cardiac catheterization. The identification of such rare vascular anatomical variations is of great importance when attempting femoral arterial or venous puncture in order to minimize unnecessary complications.

## Introduction

Across many medical specialties, there is an increasing demand for endovascular intervention. However, a thorough understanding of the vascular anatomy in the femoral region, including any anatomical variation, is essential in order to minimize unnecessary complications. The medial circumflex femoral artery (MCFA) typically presents as a major branch of the profunda femoris artery (PFA) or it can also directly originate from the common femoral artery (CFA). The MCFA is the chief source of the blood supply to the hip joint, and its anatomical variations have been described due to their clinical significance. We herein report a case of an unusual anatomical variation of the MCFA crossing anterior to the femoral vein (FV) that led to iatrogenic arteriovenous fistula (AVF) formation after cardiac catheterization.

## Case presentation

A 49-year-old man underwent catheter ablation for drug-refractory atrial fibrillation using right femoral access. A 3-French sheath was placed in the right CFA, and an 8-French sheath was placed in the right FV during the catheterization. After the procedure, he developed swelling around the puncture site, and a bruit was audible in the right groin on auscultation. An AVF was detected by color Doppler ultrasound (Figure 1). Ultrasound-guided compression was attempted but was unsuccessful. Enhanced computed tomography (CT) showed an MCFA originating from the CFA that crossed anterior to the FV and an arteriovenous communication (Figure 2).

**Figure 1:** Color Doppler ultrasonography shows the existence of an arteriovenous communication between the common femoral artery and the femoral vein. CFA, common femoral artery; FV, femoral vein

**Figure 2:** Preoperative CT images. (A) Maximum intensity projection and (B) three-dimensional reconstruction CT images showing the medial circumflex femoral artery (arrow) crossing anterior to the femoral vein and early contrast filling in the vein.

Expecting spontaneous resolution, the patient was initially treated conservatively. After six months of follow-up, the AVF did not disappear on ultrasonography, and he suffered recurrence of atrial fibrillation. Considering the risk of future cardiac complications due to sustained volume overload, surgical intervention was performed. Surgical exploration revealed a dilated MCFA that crossed anterior to the FV (Figure 3).

**Figure 3:** Intraoperative photograph showing the dilated medial circumflex femoral artery attached to the femoral vein. CFA, common femoral artery; MCFA, medial circumflex femoral artery; FV, femoral vein

The MCFA was attached to the FV, and thrill was present. Ligation of the AVF was performed. A completion angiogram demonstrated successful closure of the AVF (Figure 4).

**Figure 4:** A completion angiogram showing successful closure of the arteriovenous fistula. CFA, common femoral artery; MCFA, medial circumflex femoral artery

 The postoperative course was uneventful, and the patient was discharged on postoperative day 4.

## Discussion

An iatrogenic AVF is a potential complication of femoral arterial or venous puncture, with a rate of approximately 1% in patients undergoing cardiac catheterization [1]. Risk factors associated with AVF formation include arterial hypertension, female gender, intensified anticoagulants, and puncture of the left groin [1]. In addition, anatomical variation is a common underlying cause of puncture-related complications [2]. 

The MCFA usually arises from the PFA, but it may also originate directly from the CFA. It passes between the pectineus and psoas major and divides into its terminal branches. The deep branch of the MCFA, or the main branch, runs along the inferior border of the obturator externus towards the intertrochanteric crest [3].

Many variations in the MCFA have been described in the literature. Its anatomy has usually been described with a focus on the origin and distance to the mid-inguinal point [4,5]. The anatomical relationships between the MCFA and the lateral circumflex femoral artery have also been investigated by several groups [6-8].

In 2016, Tomaszewski et al. conducted a meta-analysis and proposed a new fivefold classification of the origin of the MCFA [5]. They found that 64.6% of MCFAs originated from the PFA, while 32.2% originated from the CFA. Among the CFA-derived MCFAs, 81.1% originated from the posteromedial aspect of the CFA as a single branch. Other variations included an origin from the superficial femoral artery (1.0%) and aplasia of the MCFA (0.4%). Accordingly, the origin of the MCFA in the present case is not very rare; however, to our knowledge, neither an anatomical variation wherein the MCFA crosses anterior to the FV nor an iatrogenic AVF between the MCFA and the FV has been previously reported.

The variations in the origin and branching pattern of the vessels of the lower limb can be explained embryologically. The MCFA develops from the arterial plexus in the ventral aspect of the thigh called the rete femorale [4]. An increase in the blood flow of the capillaries determines the persistence or elimination of capillary channels, thereby establishing the final arterial pattern. The persistence of unusual arterial channels can therefore lead to rare anatomical variations [9]. In addition, the entrance of the FV into the rete femorale can affect the positional relationship between the arteries and the FV [10].

In the present case, the cause of the AVF was assumed to be FV cannulation. The anatomical landmark technique is still used to access the FV because of the relatively constant location of the FV related to the artery at a safe entry point 2-4 cm below the level of the inguinal ligament [11]. Our case reminds us that the feasibility of landmark-based techniques is inevitably compromised by unusual anatomical variations. Similar to our case, Sahin et al. reported a rare variation of the PFA passing in front of the FV in a cadaver [10]. Other arteries at risk include the superficial epigastric, and the superficial and deep external pudendal arteries, which normally originate from the CFA and course medially.

CT angiography is a very useful method to visualize vasculature, but is not a routine test for patients who are about to undergo cardiac catheterization. In the clinical setting, ultrasound examinations are helpful for identifying any anatomical variations and the relationship among the femoral vessels. When attempting to perform an arterial puncture, having sufficient information regarding the level of the femoral bifurcation and atherosclerotic plaque is also important. Therefore, to improve the success rate of such procedures and reduce complications, ultrasound-guided vascular cannulation is recommended [11].

In a study by Kelm et al., spontaneous closure was found to occur in one-third of iatrogenic AVF cases, and cardiac volume overload was considered highly unlikely with AVF persistence [1]. However, some authors have reported high-output cardiac failure, limb edema, and limb ischemia as late complications of iatrogenic femoral AVF [12-15]. In the present case, AVF did not disappear at six months after the onset, and AVF-associated volume load could have had deleterious effects on the cardiac function in the setting of recurrent atrial fibrillation. Accordingly, we decided to perform surgical repair of the AVF in our patient, and the patient’s postoperative course was uneventful.

## Conclusions

We herein reported a rare case of an anatomical variation of the MCFA that led to iatrogenic AVF. The present case suggests that clinicians should keep in mind the possibility of unexpected vascular variations when attempting femoral arterial or venous puncture. Based on a detailed knowledge of the vascular anatomy, careful interpretation of pre-procedural CT images and the use of ultrasound imaging during vascular cannulation can improve patient safety.
